# Effects of Different Physical Exercises on Physical and Mental Health of Female College Students

**DOI:** 10.1155/2022/7812005

**Published:** 2022-03-01

**Authors:** Zhen Zhang, Hyun Joo Min

**Affiliations:** Gangneung-Wonju National University, Gangneung-si, Gangwon-do 25457, Republic of Korea

## Abstract

**Objective:**

To explore the effects of different physical exercises on the physical and mental health of female college students.

**Methods:**

This study focuses on the influence of sports intervention on the physical and mental health of female college students in H University. With the methods of literature review, investigation, measurement, experiment, and mathematical statistics, this paper discusses the influence of different physical exercises on the physical and mental health of female college students in H University.

**Results:**

The average total score of female college students' health status is 10.25, which is between the average level of L 0.34–10.72 in some universities in China. Before and after the experiment, there were significant differences in five dimensions of self-respect, balance of personality structure, natural intimacy, belief value, and ideal transcendence among all female college students in the aerobics option group. Basketball exercises have significant effects on female college students' sense of unity of body and mind, self-structure coordination, interpersonal affinity, natural affinity, belief value, self-respect, and role adaptation. Compared with before and after taking part in table tennis exercise, the mental health level of girls has significant differences in four dimensions: self-respect, balance of personality structure, interpersonal affinity, and natural affinity.

**Conclusion:**

Different physical exercises have a significant impact on female college students' physical and mental health, can improve their physical health, and have no significant impact on their social adaptability.

## 1. Introduction

With the continuous development of our society because of the needs of life and the progress of human society, many professional women appear. They have to bear some social work pressure and the important responsibility of taking care of children and families. This has also become the backbone of our society. Paying attention to the health of professional women can help maintain our social stability and build a harmonious society However, in the actual process, professional women are particularly vulnerable to various pressures from family, work, and society, resulting in varying degrees of physical and mental health problems and putting themselves in a subhealth state.

At present, people pay more and more attention to the mental health status of female college students. With the rapid development of social economy and the increasingly fierce competition, the pressure on college students is increasing, and the performance of female college students is particularly obvious and on the rise [1]. With the development of knowledge economy, women's physical and mental health has gradually become the focus of sports researchers, especially intellectual women. The most representative intellectual women are female college students in school today [2]. Female college students are the mother of society, and they should bear the important responsibility of having children in the future. The health of mothers will directly affect the health of children in the future. Therefore, it is particularly important to pay attention to women's mental health.

Female college students' physical exercise refers to the physical activities of female college students in extracurricular time, actively using various sports means and methods, in order to increase their physical quality, promote the healthy development of body and mind, enrich amateur culture, etc. [3]. This study is based on the consensus that physical exercise can improve mental health. The aim of this study is to explore the influence of different physical exercises on the mental health of female college students. At the same time, to find out whether there are differences in mental health level among different sports events, so as to provide an effective method to solve the physical and mental health problems of female college students in China and achieve the purpose of improving students' mental health.

## 2. Research Objects and Methods

### 2.1. Object of Study

Female students of grade 2019 in H University were chosen. In the aerobics group, basketball group, and table tennis group, 20 people were randomly selected, and the SCL-90 scale was distributed in the first week and the twelfth week, and students completed self-evaluation in class. A total of 150 questionnaires were distributed before and after, and 146 questionnaires were recovered with a recovery rate of 97.33%, among which 132 were valid questionnaires with an effective rate of 90.41%.

### 2.2. Research Technique

#### 2.2.1. Literature Data Method

According to the research purpose, focusing on the research on the mental health effect of physical exercise, we have consulted the works of general psychology, health psychology, sports psychology, experimental psychology, etc., and consulted dozens of related papers since the last decade. A comprehensive understanding of the current research situation in this subject area has been made, and the basic research direction has been determined.

#### 2.2.2. Interviewing Method

Interviews were conducted with subjects to understand their psychological changes.

#### 2.2.3. Questionnaire Survey Method

Through reading materials and expert interviews and using mental health scale. After logical analysis, the questionnaire form of physical exercise items was made. Through a questionnaire survey, the students' items are determined as the aerobics group, basketball group, and table tennis group.

#### 2.2.4. Measurement Method

The physiological indexes were tested before and after the experiment, including height, weight, height and body mass index (BMI), chest circumference, waist circumference, hip circumference, blood pressure (systolic and diastolic pressure), heart rate, vital capacity, step test, sitting body flexion, left and right leg longitudinal forks, and grip strength. These indicators are selected by referring to the discussion on physical indicators in Xing Wenhua's book Sports Material Selection, combining with the characteristics of aerobics and outward bound training, and seeking the opinions of relevant experts.

#### 2.2.5. Experimental Method

Three groups of female college students, aerobics group, basketball group, and table tennis group, exercise for twelve weeks under the same exercise time and frequency and use the SCL-90 scale to evaluate themselves in the first week and the twelfth week, respectively [4]. This paper makes a comparative analysis of the influence of three different exercises on the mental health level.

#### 2.2.6. Mathematical Statistics

By using the EXCEL software and SPSS 13.0 for windows software to make mathematical statistics on the survey data, it was tested whether there are significant differences between the control group and the experimental group. Mean, *t*-test, and variance analysis are mainly used.

## 3. Study Results

### 3.1. General Situation of Female College Students' Health

The results of this study show that the average total score of female college students' physical health status is 10.25, which is between the average level of 10.34 and 10.72 in some colleges and universities in China.  Table 1 shows the mental health status of the respondents.

### 3.2. Test on the Differences of Mental Health Level in the Aerobics Group before and after the Experiment

Aerobics is a kind of exercise which is popular among female friends at present. With music accompaniment and physical exercises as the basic means, aerobics as the foundation, and integrating gymnastics, dance, and music, it is one of the popular fitness methods for cultivating sentiment, enriching life, shaping the body, and entertaining. Aerobics has a more significant effect on reducing the sebum thickness of female college students' skeletons and is more conducive to improving their body shape, that is, rhythmic movement is more conducive to improving their body shape.

From Table 2, it can be seen that before and after the experiment, there are significant differences in five dimensions: self-respect, balance of personality structure, natural intimacy, belief value, and ideal transcendence, but there are no differences in four dimensions: physical and mental unity, self-structure coordination, interpersonal affinity, and role adaptation.

### 3.3. Mental Health Level and Dimensional Differences of Female College Students in the Basketball Group before and after the Experiment

According to the experimental results in Table 3, basketball exercises have significant effects on female college students' sense of unity of body and mind, self-structure coordination, interpersonal affinity, natural intimacy, belief value, self-respect, and role adaptation.

### 3.4. Mental Health Level of Girls in the Table Tennis Group before and after the Experiment

Table tennis can change people's negative personality, promote positive and healthy emotions, relieve anxiety, psychosexually transmitted diseases, and paranoia, and slowly transform narrow-minded and suspicious personality into easygoing and optimistic personality. From Table 4, it can be seen that the mental health level of girls has significant differences in four dimensions: self-respect, balance of personality structure, interpersonal affinity, and natural affinity before and after participating in the table tennis exercise.

## 4. Discussion

The differences in the mental health level between female college students in the basketball group and table tennis group after the experiment are mainly in the latitude of physical and mental unity and the latitude of role adaptation. After the experiment, the results of the comparison between the basketball group and table tennis group show that basketball is a collective sport with strong antagonism, and it is a sport that cultivates collective consciousness, unity and cooperation ability, and tenacious fighting spirit. Physical exercise is an effective method because physical exercise can not only be used as a venting means to vent the stress emotions such as worry, anxiety, and uneasiness caused by various psychological contradictions but also form harmonious interpersonal relationships and enhance self-confidence, thus balancing psychology and improving mental health [5, 6].

The research shows that there are significant differences in the mental health level of female college students in three dimensions: anxiety, paranoia, and interpersonal sensitivity. The reason is that basketball belongs to a collective antagonistic sport with great intensity, which can improve students' physical quality. In practice, both cooperation and confrontation can stimulate students' enterprising spirit and enhance their cooperative ability. Therefore, female college students' interpersonal relationship has been improved, and their anxiety and paranoia have been alleviated [7]. Studies have shown that aerobics exercise can not only relieve mental stress but also adjust tension, which also promotes the sense of balance of personality structure. During the exercise, students have a certain understanding of their physical feelings and the actual situation, which also has a certain impact on the sense of unity of body and mind. According to the interview, most of the time for these students to take part in physical exercise is after class in the afternoon, and some of the time will be during the evening classes of the community, such as participating in group sports such as dance associations and sports associations.

For female college students, mental health problems are often caused by their own factors. In this process, we can see that basketball can not only effectively compensate for the physical pressure but also effectively alleviate the real pressure problems they encounter in their daily study and life [8]. During exercise, due to muscle contraction, a lot of nutrients and oxygen are needed, so the number of contractions of the heart increases, and the amount of blood sent out every time is more than usual. At the same time, the demand for oxygen also increases, the number of breaths is more than normal, and the degree of lung expansion is also greater. The results of this experiment show that physical exercise has the most significant effect on improving the subjects' sense of self-worth, sports ability, and physical attraction. This also verifies the previous research results. Therefore, this paper holds that the reason why there are significant differences between the basketball group and table tennis group in physical and mental health level of female college students in the latitude of sense of unity of body and mind and the latitude of role adaptation.

## 5. Conclusion and Suggestion

### 5.1. Conclusion

Aerobics exercise and basketball exercise are more suitable for female college students' age characteristics and have a better effect on female college students' physical and mental health. Rhythm-type exercise with the same intensity is more effective than non-rhythm-type exercise in improving female college students' physical self-esteem. Non-rhythmic movement only has a significant effect on improving the physical condition of female college students.

Exercise intervention has played a very good role in improving some aspects of physical function of female college students in H University. If the vital capacity increases significantly, the step test value increases. It shows that exercise intervention can improve the cardiopulmonary function of the body.

Basketball exercises and table tennis exercises have different influences on female college students' physical and mental health. There are obvious differences in the mental health level between collective project and individual project. Compared with the other two events, basketball can eliminate female college students' psychological barriers such as anxiety, hostility, and sensitive interpersonal relationship. It is suggested that female college students should actively participate in physical exercise. Appropriate methods, reasonable choices, and arrangements should be adopted to motivate and guide correctly, so as to truly achieve the purpose of promoting mental health.

### 5.2. Suggestion

This study shows that taking part in physical exercise can promote the physical and mental health of female college students. Therefore, it is necessary to encourage female college students who do not have the habit of physical exercise to actively participate in physical exercise, so as to promote the continuous development of the overall physical and mental health of female college students and make contributions to improving the overall physical and mental health of college students. Therefore, basketball often plays a vital role in affecting the mental health level of female college students, which can also enhance their confidence and determination in facing life difficulties.

Female college students in H University have made significant improvements in physical and mental health after one semester's aerobics and outreach training intervention. However, because this is a means of sports intervention, if they do not insist on intervention, their physical and mental health level may fall back to the original state or worse, so it is the most crucial to cultivate students' lifelong sports awareness.

Female college students are in poor physical and mental health, and the amount of physical exercise is too small. Therefore, it is suggested that H University should strengthen the mental health education for college students in women's colleges, especially the education that physical exercise can improve physical and mental health and adopt practical implementation measures. For example, increasing and rationally using venues and equipment can ensure the amount of physical exercise for female college students and improve their mental health.

## Figures and Tables

**Table 1:** Descriptive statistics of female college students' physical and mental health.

	Quantity	Minimum value	Maximum value	Average score	Standard deviation
Good health	60	0	45	10.25	7.85

**Table 2:** Test on the differences of mental health level in the aerobics group before and after the experiment.

Dimension	Before the experiment (*n* = 20)	After the experiment (*n* = 20)	*t*	*p* value
Sense of unity of mind and body	15.22 ± 4.28	15.69 ± 2.01	−1.52	0.010
Sense of self-respect	21.04 ± 2.48	21.82 ± 2.01	−2.88	0.053
Sense of balance of personality structure	16.93 ± 3.23	17.24 ± 3.02	−1.72	0.074
Self-structure coordination	14.86 ± 2.91	14.99 ± 2.01	−0.25	0.006
Interpersonal affinity	23.61 ± 7.66	23.71 ± 6.88	−4.85	0.052
Role adaptation	10.28 ± 1.56	10.56 ± 1.73	−3.96	0.071
Natural intimacy	11.42 ± 2.19	11.93 ± 1.53	−4.11	0.082
Sense of belief value	17.83 ± 2.01	18.24 ± 2.41	−2.82	0.041
Ideal transcendence	18.25 ± 2.14	18.69 ± 2.33	−6.88	0.063

**Table 3:** Comparison of scores of female college students in the basketball group before and after the experiment.

Dimension	Before the experiment (*n* = 20)	After the experiment (*n* = 20)	*t*	*p* value
Sense of unity of mind and body	12.28 ± 4.02	13.01 ± 2.11	−2.17	0.006
Sense of self-respect	17.02 ± 3.27	18.11 ± 3.26	−5.26	0.108
Sense of balance of personality structure	15.26 ± 2.06	16.93 ± 2.71	−1.19	0.072
Self-structure coordination	10.27 ± 1.02	10.96 ± 1.24	−5.58	0.101
Interpersonal affinity	2.33 ± 5.02	2.63 ± 4.21	−1.74	0.032
Role adaptation	11.62 ± 3.71	12.80 ± 3.07	−5.32	0.062
Natural intimacy	16.28 ± 2.66	17.88 ± 2.53	−4.21	0.071
Sense of belief value	13.82 ± 2.81	14.82 ± 2.62	−3.82	0.006
Ideal transcendence	19.62 ± 4.18	20.19 ± 4.28	−4.66	0.203

**Table 4:** A test on the differences of mental health level of girls in the table tennis group before and after the experiment.

Dimension	Before the experiment (*n* = 20)	After the experiment (*n* = 20)	*t*	*p* value
Sense of unity of mind and body	14.22 ± 4.21	14.27 ± 4.28	−1.25	<0.001
Sense of self-respect	20.11 ± 2.16	21.05 ± 2.03	−6.88	0.005
Sense of balance of personality structure	13.20 ± 2.93	14.62 ± 3.14	−4.21	0.021
Self-structure coordination	14.82 ± 3.81	15.93 ± 3.30	−3.08	0.301
Interpersonal affinity	11.08 ± 2.17	12.82 ± 2.41	−1.72	0.003
Role adaptation	22.01 ± 1.83	22.24 ± 2.42	−3.86	0.028
Natural intimacy	18.52 ± 2.11	18.93 ± 2.37	−4.21	0.064
Sense of belief value	14.20 ± 2.16	14.58 ± 2.88	−5.66	0.082
Ideal transcendence	13.07 ± 2.50	13.73 ± 2.71	−7.08	0.063

## Data Availability

The data used to support the findings of this study are included within the article.
